The article "Identification of novel natural inhibitors targeting AKT Serine/Threonine Kinase 1 (AKT1) by computational study" was retracted in 2026. Reason: concerns about the authorship.

# Identification of novel natural inhibitors targeting AKT Serine/Threonine Kinase 1 (AKT1) by computational study

**DOI:** 10.1080/21655979.2021.2011631

**Published:** 2022-05-21

**Authors:** Sheng Zhong, Yuanyuan Hou, Zhiyun Zhang, Zhen Guo, Wenzhuo Yang, Gaojing Dou, Xiaye Lv, Xinhui Wang, Junliang Ge, Bo Wu, Xuefeng Pan, Hongyu Wang, Qunying Yang, Yonggao Mou

**Affiliations:** a Neurosurgery and Neuro-Oncology Department, Sun Yat-Sen University Cancer Center, State Key Laboratory of Oncology in South China, Collaborative Innovation Center for Cancer Medicine, Guangzhou, China; b Clinical College, Jilin University, Changchun, China; c Department of Breast surgery, the First Bethune Hospital of Jilin University, Changchun, China; d Department of Hematology, the First Clinical Medical School of Lanzhou University, Lanzhou, Gansu, China; e Department of Oncology, the First Hospital of Jilin University, Changchun, China; f Department of Orthopaedics, the First Bethune Hospital of Jilin University, Changchun, China; g Department of Obstetrics, the First Bethune Hospital of Jilin University, Changchun, China

**Keywords:** AKT1, ipatasertib, drug treatment, discovery studio, virtual screening, CCK8, ELISA

## Abstract

Despite great progress, the current cancer treatments often have obvious toxicity and side effects. and a poor prognosis (some patients). One of the reasons for the poor prognosis is that certain enzymes prevent anticancer drugs from killing tumor cells. AKT1 is involved in regulating PI3K/AKT/mTOR, a tumor-generating pathway. Ipatasertib, a highly selective inhibitor of AKT1, is widely used in the treatment of tumors. In this study, many structural and biochemical methodswere used to find better AKT1(Threonine Kinase 1) inhibitors, which laid a foundation for the further development of AKT1 inhibitors and provided new drugs for the treatment of tumors. ZINC15 database and Discovery Studio 4.5, a computer-aided drug screening software with many modules (LibDock for virtual screening, ADME (Absorption, Distribution, Metabolism, Excretion) and TOPKAT (toxicity prediction module) for the toxicity and properties analysis, and MD simulation for stability prediction), were employed. CCK8 assay, ELISA assay genicity and higher tolerance to cytochrome P4502D6. MD simulations indicated they could bind with AKT1 stably in the natural environment. The cell experiment and specific assay for AKT1 inhibition showed they could inhibit the proliferation and AKT1 expression of MG63 cells (Osteosarcoma cells). Moreover, these novel compounds with structural modifications can be potential contributors that lead to further rational drug design for targeting AKT1.

**Abbreviation**AKT1, AKT Serine/Threonine Kinase 1; ADME, absorption, distribution, metabolism, excretion; TOPKAT, toxicity prediction by Computer assisted technology; CCK8, Cell Counting Kit 8; ELISA, Enzyme-linked immunosorbent assay; CYP2D6, cytochrome P4502D6 inhibition; GBM, Glioblastoma; AGC kinase, protein kinase A, G, and C families (PKA, PKC, PKG); PKB, protein kinase B; PAM pathway, PI3K/AKT/mTOR pathway; OS, overall survival; PFS, progression-free survival; LD50, lethal dose half in rats; LOAEL, lowest observed adverse effect level; NPT, normal pressure and temperature; PME, particle mesh Ewald; LINCS, linear constraint solver; RMSD, root-mean-square deviation; BBB, blood–brain barrier; DS, Discovery Studio; DTP, Developmental toxicity potential; PPB, Plasma protein binding; MTD, Maximum Tolerated Dosage; AB, Aerobic Biodegradability; NTP, US. National Toxicology Program; DTP, developmental toxicity potential.

## Highlights

- ZINC000049872065 and ZINC000021992902 were selected as safe drug candidates.
- Candidate compounds played an important role in AKT1 inhibitor development.
- A list of drug candidates with pharmacologic properties was provided.
- This study contributed to AKT1 or other proteins in medication design and improvement.

## Introduction

Cancer is the most fatal disease in the twenty-first century and becomes the second leading cause of death in humans. Osteosarcoma is the most common primary malignant bone tumor in children and adolescents. The onset peak occurred during the growth spurt of adolescence [1,2]. Due to micrometastatic spread, radical surgery alone rarely results in cure. For decades, there has been little progress in the treatment of osteosarcoma and no significant improvement in prognosis [3]. Glioblastoma (GBM) is a rare tumor and one of the most challenging malignancies in all of oncology. Although there have been advances in the treatment of GBM, no encouraging results have been observed in general. Patients who are diagnosed with these tumors often have a poor prognosis and poor quality of life as the disease progresses. In addition, GBM exhibits large intertumor and intra – tumor heterogeneity, complicating the development of effective therapeutic strategies^4^[5][6]. Lung cancer is the leading cause of cancer-related death worldwide, and 5-year survival rates vary between 4% and 17%, depending on stage and region [7]. Some patients were still receiving conventional chemotherapy, but the effect was moderate. Primary or secondary drug resistance ultimately leads to treatment failure in all patients with advanced disease [8]. In recent years, the treatment of cancer has developed a lot including surgery, radiotherapy, chemotherapy and immunotherapy [9]. However, current treatments have many adverse effects. Surgical resection is an important way to treat cancer, and in most cases, it can effectively relieve patients’ symptoms. However, increasing evidence suggests that surgical excision may enhance the metastatic seeding of tumor cells [10]. For example, gastric adenocarcinoma is the fifth most common cancer and the third most deadly cancer globally. Surgery is the only chance of cure, but relapse is common even with complete resection [11]. Radiation not only can reduce the absolute risk of dying of breast cancer by a few percentage points for the right patient but also it can lead to a second cancer or heart disease decades later [12]. Toxicity during chemotherapy in patients with advanced ovarian cancer is common and varied [13]. Although immunotherapy is generally more effective and better tolerated than traditional and targeted therapies, many patients have an innate or acquired resistance to immunotherapy [14]. Determining the dominant drivers of cancer immunity is a major challenge of immunotherapy [15]. Furthermore, one of the long-term side effects of chemotherapy is the risk of developing other cancers [16]. Besides, even though the treatments are developing rapidly, the five-year survival rates of lung cancer (15%), liver cancer (7%) and glioblastoma (5%) are still very low [16,17]. There is still a lack of efforts to improve the effectiveness of treatment. One of the reasons for the poor prognosis is that certain enzymes in the body prevent cancer drugs from killing tumor cells through certain mechanisms. So, we tried to find drugs in the ZINC database that could inhibit those enzymes and thus eliminate their inhibition of cancer drugs.

AKT is a member of the AGC kinase (protein kinase A, G, and C families (PKA, PKC, PKG)) family, which is essentially a threonine/serine protein kinase, and is also widely known as protein kinase B (PKB). As the core of PAM (PI3K/AKT/mTOR) pathway, a well-known pathway that regulates tumorigenesis, once AKT is activated, the polyploidy, hepatocellular carcinoma and mitotic arrest can be promoted by it [18]. However, if AKT is overactivated, it can cause excessive depletion of hematopoietic stem cells in mice and induce leukemia [19]. AKT1, AKT2, and AKT3 constitute the AKT family. AKT1 is an important factor in tumor growth, and AKT2 plays an vital role in the distant metastasis of tumors. However, no significant progress has been made in the study of AKT3, and it has only been found to have an important role in triple-negative breast cancer.

AKT1 affected many functions of tumor cells, including cell proliferation, apoptosis, migration, and transcription [20,21]. Activation or abnormal expression of AKT1 is widely observed in pancreatic, lung, ovarian, and lung cancers [22]. Therefore, effective treatment with AKT1 inhibitors is necessary. Recently, however, some studies have found some compounds that can inhibit AKT1, such as Ipatasertib, a highly selective inhibitor targeting AKT1 [23]. It is currently available to treat cancer as a single targeted agent or in combination with other cancer therapies [24]. Ipatasertib is currently available in combination or alone. Results of a double-blind phase study of prostate cancer patients treated with Ipatasertib in combination with prednisolone/prednisolone and abirone showed that Ipatasertib in combination with prednisolone/prednisolone and abirone extended the overall survival (OS) and progression-free survival (PFS) in patients with PTEN-deficient metastatic removal. Therefore, the purpose of this study is to screen out more effective AKT1 inhibitory drug candidates than Ipatasertib from the natural compound database of ZINC15.

Natural compounds have become an important source of the pharmaceutical industry. By certain structural modification of natural compounds, we can obtain drugs with good pharmacological properties in many aspects [25,26]. In recent years, the progress of research on AKT1 inhibitory drugs has been slow. In order to screen out new potential AKT1 inhibitory drugs, we used a series of structural biological and chemical methods (including virtual screening, molecular docking, etc.) for virtual screening. Besides, a CCK8 assay and ELISA were performed to verify the effect of potential compounds. This study laid a foundation for the further development of AKT1-targeted inhibitory drugs, which will promote its development to a large extent.

## Methods

### Discovery studio software and ligand library

Discovery Studio 4.5 has become an important software in the field of molecular modeling and life science research after several iterations. Discovery Studio 4.5 provides researchers with tools for protein optimization, modeling, and drug design through the application of protein structure and protein structure biological computation. In recent years, the pharmaceutical industry has used the software to screen and refine a large number of potential drug candidates from natural compound databases and other drug databases. Multiple modules of Discovery Studio 4.5 (LiDock, CDOCKER, ADME, etc.) were used in this study to conduct drug screening. For virtual screening, LibDock was employed; CDOCKER was used for docking research; ADME was used to analyze pharmacological properties. The ZINC15 database is a free database of commercially available compounds provided by the Irwin and Shoichet Laboratories, Department of Pharmaceutical Chemistry, University of California, San Francisco (San Francisco, California, USA) [27–29].

### Use LibDock for structure-based virtual filtering

In order to virtually screen compounds with potential inhibitory effects on AKT1, the LibDock module of Discovery Studio 4.5 was used in this study and the ligand-binding pocket of AKT1 was selected as the binding site [30]. LibDock calculates protein hotspots that can further be used to align the ligands to form favorable interactions using a grid placed at the binding site and polar probes and nonpolar probes. In order to perform ligand minimization, CHARMM force field and the Smart Minimizer algorithm were employed. After minimization, all ligand poses were ranked based on the ligand score. The 2.0 Å crystal structure of human AKT1 (Figure 1) and the inhibitor Ipatasertib were downloaded from the Protein Data Bank and imported to the working circumstance of LibDock. The prepared protein was obtained by a 2000-step minimization process with a root-mean-square gradient deviation of 12.277 and a final root-mean-square gradient of 0.690. Binding sites were defined by the prepared proteins. To perform virtual screening, LibDock docked all the prepared ligands at the defined active site which was generated by using the ligands of AKT1 binding position. All candidate compounds were ranked according to the LibDock score [31–33].

**Figure 1.** Molecular structure of AKT1. (a) Initial molecular structure. (b) Molecular structure with binding area of its surface. Blue represents positive charge, and red represents negative charge.

### ADME (Absorption, Distribution, Metabolism, and Excretion) and Toxicity Prediction

To calculate the absorption, distribution, metabolism, and excretion (ADME) of selected compounds, including their blood–brain barrier penetration, aqueous solubility cytochrome, hepatotoxicity, plasma protein binding levels, and P-450 2D6 (CYP2D6) inhibition, ADME and TOPKAT modules of Discovery Studio 4.5 were selected in this study. To fully analyze pharmacological properties and further screen-appropriate AKT1 candidates, the TOPKAT module was employed to calculate Ames mutagenicity, rodent carcinogenicity under the US. National Toxicology Program, oral lethal dose half in rats (LD50), potential for developmental toxicity, and lowest chronic oral observed adverse effect level (LOAEL).

### Molecular dynamics simulation

The optimal structural conformation of the ligand-AKT1 complexes were obtained through the previous molecular docking procedures. Next, the optimal structural conformation of the ligand – AKT1 was submitted to the molecular dynamics simulation module [34,35]. The ligand-receptor complex was put into an orthorhombic box and solvated with an explicit periodic boundary solvation water model. In order to simulate the physiological environment, sodium chloride was added to the system with an ionic strength of 0.145. Then the system was subjected to the CHARMM force field that was used for ligand parameterization based on analogy [36,37]. For the system, the following simulation protocols were applied: 1000 steps of minimization by steepest descent and conjugate gradient; 250ps-equilibration simulations in temperature of 300 K (slowly driven from initial temperature of 50 K for 200ps) and normal pressure ensemble; 110ps-MD simulation (production module) under NPT (normal pressure and temperature). The particle mesh Ewald (PME) algorithm was used to calculate long-range electrostatics, and the linear constraint solver (LINCS) algorithm was adapted to fix all bonds involving hydrogen. With initial complex setting as a reference, a trajectory was determined for root-mean-square deviation (RMSD), potential energy, and structural characteristics through the Discovery Studio 4.5 analysis trajectory protocol in Discovery Studio 4.5.

### Experiment to verify the therapeutic effect of the two selected compounds on the viability of MG63 cells and AKT1 expression in MG63 cells

#### Cell culture

In this study, MG63 cell lines (osteosarcoma cell lines) were cultured in high-glucose DMEM medium containing 10% fetal bovine serum at 37°C and 5% CO2 until the cells covered the bottom of the flask. After one cell passage, the cells were further cultured. Cells in logarithmic growth phase were selected for cell experiment and cell morphology was observed under light microscope (Zeiss, Axiovert 200, Germany).

#### CCK8 assay

MG63 cells were seeded into 96-well plates at a density of 5 × 103/well, and each group had three duplicate wells. After 24 h, Ipatasertib, Andropanoside (ZINC000049872065) and Neoandrographolide (ZINC000021992902) were added into 96-well plates with increasing drug concentrations and then cultured in 5%CO2 at 37°C for 72 h. Each drug was divided into 13 groups with dosage of 0.1 μmol/L, 0.25 μmol/L, 0.5 μmol/L, 0.75 μmol/L, 1 μmol/L, 2.5 μmol/L, 5 μmol/L, 7.5 μmol/L, 10 μmol/L, 25 μmol/L, 50 μmol/L, 75 μmol/L and 100 μmol/L. Add 100 μL test solution (including 10 μL CCK8 + 90 μL DMEM medium) to each well and incubate at 37°C for 1 h. The absorbance of the solution at 450 nm was determined by enzyme plate analyzer.

#### Detection of AKT1

The cell culture and grouping were the same as mentioned above. The operation was carried out according to the instructions of the ELISA detection kit, and the AKT1 expression of MG63 cells was measured.

#### Specific assay for AKT1 inhibition by selected compounds

The cell culture was the same as mentioned above. The supernatant of cell culture was obtained, and MG63 cells were seeded into 6-well plate cells for culture. After 24 h, andropanoside (ZINC000049872065) and neoandrographolide (ZINC000021992902) were added into 6-well plates with increasing drug concentrations and then cultured in 5% CO2 at 37°C for 72 h. Then, the ELISA detection kit was used to detect the expression of AKT1.

## Results

The current treatment of cancer has many toxic and side effects, and the prognosis of patients is still poor after treatment. One of the main reasons for the poor prognosis is that certain enzymes in the body work through some mechanism to prevent anticancer drugs from killing tumor cells. Among them, AKT1 is abnormally activated and expressed in a variety of cancers, and the use of AKT1 inhibitor Ipatasertib can effectively inhibit tumor proliferation and metastasis. But Ipatasertib has irreversible side effects. Therefore, our goal is to screen out more effective AKT1 inhibitor candidates than Ipatasertib from the ZINC15 natural compound database to provide more ideas for the treatment of cancer. In this study, we applied the Libdock to initially screen 17,931 commercially available drugs in the ZINC database, and selected the top 20 with the highest Libdock scores. Through ADME, TOPKAT, CDOCKER, and Molecular Dynamics simulation, we selected two optimal drugs: andropanoside (ZINC000049872065) and neoandrographolide (ZINC000021992902). Finally, CCK8 and ELISA assays were used to verify the therapeutic effect of the two compounds on the viability of MG63 cells and the expression of AKT1 in MG63 cells. Under the experimental conditions set by us, both drugs can completely inhibit the expression of AKT1 at about 10 µmol/L.

### Virtual screening of natural products database against AKT1

In order to perform virtual screening, we selected ligand-binding pocket region as the reference site, one of the regulatory sites of AKT1 Table 1. In this study, AKT1 was selected as the receptor protein, and 17,931 purchasable natural product molecules were screened from the ZINC15 database as ligands for further screening. The results of LibDock indicated that 7764 natural molecules could dock with AKT1 and the top 20 molecules with higher scores were selected for further screening and study.

**Table 1.** Top 20 ranked compounds with higher libdock scores than Ipatasertib

Number	Compounds	Libdock Score	Molecular Formula	Chemical Structure
1	ZINC000014951634	168.745	C32H37N5O5	
2	ZINC000014951658	166.943	C34H38N6O5	
3	ZINC000028968101	145.408	C33H34O7	
4	ZINC000049872065	141.722	C26H40O9	
5	ZINC000002509755	140.459	C23H24N2O4	
6	ZINC000015122022	140.179	C25H28O6	
7	ZINC000002528486	139.207	C23H24N2O4	
8	ZINC000001531664	138.246	C32H22O10	
9	ZINC000013328774	137.404	C23H22O10	
10	ZINC000021992902	135.637	C26H40O8	
11	ZINC000030725991	134.058	C36H38N2O6	
12	ZINC000002526388	133.986	C24H26N2O5	
13	ZINC000008844372	133.522	C22H22O9	
14	ZINC000013378636	133.393	C25H28O5	
15	ZINC000073280937	132.993	C35H37NO8	
16	ZINC000030730842	132.136	C16H23N5O6	
17	ZINC000006528354	132.056	C20H22O6	
18	ZINC000044281738	131.796	C34H26O8	
19	ZINC000028882432	131.625	C26H32O11	
20	ZINC000008214697	131.398	C27H50O6	

### ADME and toxicity prediction

The pharmacologic properties of the candidate drugs (the top 20 compounds) and reference drugs, Ipatasertib, were analyzed and predicted using the ADME module of Discovery Studio 4.5 (Table 2). The results of the aqueous solubility prediction part showed that most of the compounds had a good aqueous solubility (the prediction was defined in 25°C). For hepatotoxicity and plasma protein-binding properties (PPB) part, 8 compounds were nontoxic and 10 compounds had weak absorption. Besides, four compounds had a medium BBB (blood–brain barrier) level, while the other compounds were undefined and 70% of the compounds were predicted to be non-inhibitors with P450 2D6 (CYP2D6). As for human intestinal absorption prediction, four compounds had a good human intestinal absorption as the reference drug had.

**Table 2.** ADME(Absorption, Distribution, Metabolism, and Excretion) properties of compounds

Number	Compounds	Solubility Level	BBB Level	CYP2D6	Hepatotoxicity	Absorption Level	PPB Level
1	ZINC000014951634	3	4	0	0	3	0
2	ZINC000014951658	3	4	0	0	3	0
3	ZINC000028968101	1	4	1	1	3	1
4	ZINC000049872065	3	4	0	0	2	0
5	ZINC000002509755	2	2	1	1	0	1
6	ZINC000015122022	2	4	1	0	2	1
7	ZINC000002528486	2	2	1	1	0	1
8	ZINC000001531664	2	4	0	1	3	0
9	ZINC000013328774	3	4	0	1	3	0
10	ZINC000021992902	3	4	0	0	1	0
11	ZINC000030725991	0	4	0	1	2	0
12	ZINC000002526388	2	4	1	1	0	1
13	ZINC000008844372	3	4	0	1	1	0
14	ZINC000013378636	2	4	1	0	2	1
15	ZINC000073280937	2	4	0	1	2	1
16	ZINC000030730842	4	4	0	1	3	0
17	ZINC000006528354	3	2	0	1	0	1
18	ZINC000044281738	0	4	0	1	3	1
19	ZINC000028882432	3	4	0	0	3	0
20	ZINC000008214697	2	4	0	0	3	1
21	Ipatasertib	2	2	0	0	0	0

BBB, blood-brain barrier; CYP2D6, cytochrome P-450 2D6; PPB, plasma protein binding.

Solubility level: 0, extremely low; 1, very low, but possible; 2, low; 3, good.

BBB level: 0, very high penetrant; 1, high; 2, medium; 3, low; 4, undefined.

CYP2D6 level: 0, noninhibitor; 1, inhibitor.

Hepatotoxicity: 0, nontoxic; 1, toxic.

Human-intestinal absorption level: 0, good; 1, moderate; 2, poor; 3, very poor.

PPB: 0, absorbent weak; 1, absorbent strong.

Drug safety screening was a crucial part of this study. In order to evaluate the toxicity of the top 20 candidate compounds and Ipatasertib and ensure the safety of them, the TOPKAT module of Discovery Studio was selected in this study to evaluate and analyze a number of toxicity index parameters (Table 1 and Table 3). The software analysis results showed that 7 compounds had no developmental toxicity potential and there were 12 non-mutagenic compounds, while the rodent carcinogenicity of Ipatasertib was high. Considering ZINC000049872065 and ZINC000021992902 were less carcinogenic, non-hepatotoxic, and non-CYP2D6 inhibitors, we selected these two compounds as safe drugs for the following study (Figure 2).

**Table 3.** Toxicities of compounds

Number	Compounds	Mouse NTP		Rat NTP		Ames	DTP
		Female	Male	Female	Male		
1	ZINC000014951634	0.089	0	1	0	0	1
2	ZINC000014951658	1	0	1	0	0	1
3	ZINC000028968101	1	0.021	0.06	0.997	1	1
4	ZINC000049872065	0.353	0	0.752	0.006	0	0
5	ZINC000002509755	0.603	0.001	0	0.535	0.996	0.019
6	ZINC000015122022	0	1	1	0	1	1
7	ZINC000002528486	0.603	0.001	0	0.535	0.996	0.019
8	ZINC000001531664	0.999	1	0	1	0	1
9	ZINC000013328774	0.865	1	1	1	0.674	1
10	ZINC000021992902	0.198	0	0.033	0.251	0	0
11	ZINC000030725991	0	0	0.163	1	0	1
12	ZINC000002526388	0.999	0.041	0	0.999	0.999	0.745
13	ZINC000008844372	1	1	1	1	0	1
14	ZINC000013378636	0	1	1	0	1	1
15	ZINC000073280937	0.312	1	0	0.185	0	1
16	ZINC000030730842	1	1	0.001	0	1	0
17	ZINC000006528354	0.151	0	1	0	0.002	1
18	ZINC000044281738	0	0	1	0	0.007	0
19	ZINC000028882432	0.081	1	0	0.987	0	1
20	ZINC000008214697	0	0.003	0	1	0	0
21	Ipatasertib	1	0	0.985	0	0	1

NTP, U.S. National Toxicology Program; DTP, developmental toxicity potential.

NTP<0.3 (noncarcinogen); >0.8 (carcinogen).

Ames<0.3 (nonmutagen); >0.8 (mutagen).

DTP<0.3 (nontoxic); >0.8 (toxic).

**Figure 2.** Structures of novel compounds (a, b) and (c)Ipatasertib selected from virtual screening.

### Analysis of ligand binding

The ligand-binding mechanisms of these two chosen compounds with AKT1 were studied by CDOCKER, a module of Discovery Studio 4.5, which can dock these two into the structure of AKT1. The CDOCKER results showed that the CDOCKER potential energy of the reference drug Ipatasertib was significantly higher than that of the candidate compounds of ZINC000049872065 and ZINC000021992902, which indicated that the binding affinity between the candidate compounds and AKT1 was higher than that of the reference drug (Table 4). The study of π-related interactions and hydrogen bonds was also performed (Figures 3 and 4). The docking results of CDOCKER showed that 12 pairs of hydrogen bonds were formed between AKT1 and ZINC000049872065, while 10 pairs of hydrogen bonds were formed between AKT1 and ZINC000021992902. At the same time, we also used CDOCKER to study the hydrogen bonds and π-related interactions between Ipatasertib and AKT1, the results showed that there were 5 pairs of hydrogen bonds and one pair of π-related interactions between Ipatasertib and AKT1 (Tables 5 and 6).

**Table 4.** CDOCKER potential energy of compounds with AKT1 under CHARMM force field

Compounds	-CDOCKER Potential Energy (kcal/mol)
ZINC000049872065	58.7801
ZINC000021992902	56.4843
Ipatasertib	49.9388

**Table 5.** Hydrogen bond interaction parameters for each compound with AKT1

Receptor	Compound	Donor Atom	Receptor Atom	Distances(Å)
3MV5	ZINC000049872065	GLY159:HN	ZINC000049872065:O22	2.64
		LYS179:HZ1	ZINC000049872065:O35	1.88
		GLY294:HN	ZINC000049872065:O35	2.85
		ZINC000049872065:H52	THR291:OG1	2.53
		ZINC000049872065:H54	GLU234:OE1	1.97
		ZINC000049872065:H56	LEU156:O	2.36
		GLY157:HA1	ZINC000049872065:O18	2.31
		GLY157:HA2	ZINC000049872065:O18	2.45
		ZINC000049872065:H49	GLU234:OE1	2.41
		ZINC000049872065:H51	ASP292:OD2	2.48
		ZINC000049872065:H55	GLU234:OE1	2.23
		ZINC000049872065:H75	GLU191:OE1	2.63
	ZINC000021992902	GLY294:HN	ZINC000021992902:O34	2.74
		ZINC000021992902:H51	ASP292:OD2	2.24
		ZINC000021992902:H53	GLU234:OE1	1.96
		ZINC000021992902:H55	LEU156:O	2.52
		GLY157:HA1	ZINC000021992902:O18	2.32
		GLY157:HA2	ZINC000021992902:O18	2.36
		ZINC000021992902:H48	GLU234:OE1	2.38
		ZINC000021992902:H49	ASP292:OD2	2.72
		ZINC000021992902:H54	GLU234:OE1	2.29
		ZINC000021992902:H74	GLU191:OE1	3.08
	Ipatasertib	LYS276:HZ1	Molecule:O8	1.69
		Molecule:H56	GLU234:OE1	2.08
		GLY157:HA1	Molecule:N16	2.91
		Molecule:H44	ASN279:OD1	2.83
		Molecule:H46	ASP292:OD2	2.47

**Table 6.** π-Related Interaction Parameters for Each Compound with AKT1

Receptor	Compound	Donor Atom	Receptor Atom	Distances(Å)
3MV5	ZINC000049872065	A:PHE161	ZINC000049872065	4.48
	ZINC000021992902	/	/	/
	Ipatasertib	Molecule:C20	A:VAL164	4.45

**Figure 3.** Schematic drawing of interactions between ligands and AKT1. The surface of the binding areas was added. Blue represents positive charge; red represents negative charge; and ligands are shown in sticks, with the structure around the ligand -receptor junction shown in thinner sticks. (a) ZINC000049872065-AKT1 complex. (b)ZINC000021992902-AKT1 complex. (c) Ipatasertib-AKT1 complex.

**Figure 4.** Schematic of intermolecular interaction of the predicted binding modes of (a) ZINC000049872065 withAKT1, (b) ZINC000021992902 with AKT1, and (c) Ipatasertib with AKT1.

### Molecular dynamics simulation

The original conformation required for the molecular dynamics simulation experiments was obtained through the CDOCKER module of Discovery Studio 4.5. After a certain period of time, both the potential energy and RMSD of these compounds can reach a relatively stable and balanced state at 20ps (the trajectory curves of potential energy and RMSD are shown in Figure 5). Based on the results of molecular dynamics experiments, this study concluded that ZINC000049872065 and ZINC000021992902 could combine with AKT1 in the natural environment as a complex and exist stably.

**Figure 5.** Results of molecular dynamics simulation of two compounds. (a) Potential energy (b) Average backbone RMSD.

### Statistical analysis

MG63 cells were treated with ipatasertib, andropanoside (ZINC000049872065), and neoandrographolide (ZINC000021992902) for 72 hours. Then the cell viability was detected by the CCK8 kit. The results showed that Ipatasertib, Andropanoside and Neoandrographolide had an inhibitory effect on the proliferation of MG63 cells compared with the blank control group. The cell viability of Ipatasertib, Andropanoside and Neoandrographolide group was smaller than that of blank group, and the inhibitory effect of Andropanoside and Neoandrographolide group on the proliferation of MG63 cells was stronger than that of Ipatasertib group (Figure 6 and Figure 7).

**Figure 6.** Andropanoside group of CCK8 assay: Cellular viability of MG63 cells.

**Figure 7.** Neoandrographolide group of CCK8 assay: Cellular viability of MG63 cells.

Additionally, the level of AKT1 secretions in Ipatasertib, andropanoside, and neoandrographolide group were lower than that in blank group, and the level of AKT1 secretions in Andropanoside and Neoandrographolide group were lower than that in Ipatasertib group. It is suggested that the Ipatasertib, andropanoside, and neoandrographolide group has an inhibitory effect on the level of AKT1 secretion of MG63 cells compared with the blank group (Figure 8).

**Figure 8.** Detection of AKT1 expression in MG63 cells by ELISA.

Finally, 13 groups of two selected compounds at different concentrations were used to detect the degree of inhibition of AKT1 expression at different concentrations. The results showed that with the increase in drug concentration, the inhibition degree of AKT1 was stronger (Figure 9). In addition, the experimental results showed that under the experimental conditions set by us, the two drugs could completely inhibit the expression of AKT1 at about 10 µmol/L.

**Figure 9.** Detection of AKT1 expression in MG63 cells in different concentrations of drugs by ELISA.

## Discussion

In recent years, the development of new AKT inhibitors for clinical application and their combination with different anticancer drugs to improve the therapeutic effect have become a research hotspot in the field of antineoplastic drugs.

Previous studies on inhibitors of AKT1 have shown that AKT1 plays an important role in tumorigenesis regulation. Although a lot of progress has been made in the research of targeted AKT1 therapy, the therapeutic effect of AKT1 inhibitors is not satisfactory [38–44]. Hence, to screen more compounds targeting AKT1 is urgent. In this research, ipatasertib was selected as a reference drug in this study. Ipatasertib is a highly selective ATP-competitive small-molecule AKT inhibitor that showed activity in a broad range of cancer types, including prostate, breast, ovarian, colorectal, and non-small-cell lung cancers [45].

In order to screen out more potential drug candidates that can inhibit AKT1, four modules of the software (Discovery Studio 4.5), including LibDock, ADME/TOPKAT, CDOCKER, and Molecular Dynamics Simulation, were employed to screen and analyze the structural and biological properties of novel potential compounds, respectively.

For the purpose of preliminary screening of 17,931 commercially available drugs, the LibDock module was applied, and 7764 drugs with higher LibDock scores were preliminarily screened from the ZINC15 database. The higher LibDock score was, the better the energy optimization of this molecule was, and the more stable the conformation would be, which means that the higher LibDock score, the higher binding affinity with AKT1. During the screening of drug candidates, the LibDock score of the reference drug, Ipatasertib, was also evaluated and ranked by the software. The results showed that the LibDock score of many drugs was higher than that of the reference drug. We selected the top 20 compounds for further screening.

Although having a better affinity binding to AKT1 than Ipatasertib may partially account for their advantage, it is far from sufficient. The toxicity properties of these selected compounds and whether their pharmacological properties are conducive to their role in clinical use also need to be considered. Results of prediction of ADME and toxicity properties showed that ZINC000049872065 and ZINC000021992902 were more suitable for screening as potential drug candidates because their water solubility and absorption level were superior to those of the other 18 compounds. In addition, these two compounds showed less rodent carcinogenicity, developmental toxicity, and Ames mutagenicity than other compounds, and neither of them was hepatotoxic because they were non-cytochrome P450 2D6 (CYP2D6) inhibitors. Therefore, based on the safety aspect, they have great potential for future clinical use. Although the other drugs on the list are toxic, they also have the potential to be used in future studies by adding specific groups and atoms to make them less toxic. Considering all the above properties, these two compounds were more suitable for screening as potential AKT1 inhibitors.

However, good binding affinity and safety were only the basic properties of targeted therapy drugs. In order to reflect the superiority of candidate compounds and increase the possibility of their future clinical application, CDOCKER module, Molecular Dynamic Simulation module, and cell experiments (CCK8 assay, ELISA in vitro and Specific assay for AKT1 inhibition) were used to further study and analyze the docking mechanism and chemical bonds between the two candidate compounds and AKT1, their stability in the natural environment and the effectiveness of the compounds. CDOCKER module computation and molecular structure inspection showed that CDOCKER interaction energy of Ipatasertib was higher than these 2 compounds and there were more chemical bonds formed between them and AKT1 in comparison with Ipatasertib. Based on the results, we were able to infer that these two compounds bound more closely to AKT1 during targeted therapy than Ipatasertib, resulting in stronger inhibition of AKT1 activity and a more powerful killing effect on tumors.

Finally, Molecular Dynamic Simulation indicated that these two compounds can combine with AKT1 stably in the natural environment to exert their inhibitory effect, and cell experiments also showed that these two compounds have stronger inhibitory effect than Ipatasertib. Based on the current study, our future research will focus on further modification and refinement of the compounds to make the ligand bind to the receptor more firmly.

In previous studies, our research methods have been widely used, such as the screening of CD13 natural inhibitors [46], bacopa monnieri in the treatment of Alzheimer’s Disease [47], novel inhibitors against β-lactamase CTX-m-152 [48], MCL-1 inhibitors [49], etc., using the same or similar research methods as ours. The drugs screened by this method showed good properties and efficacy. There are many types of AKT1 inhibitors. Capivasertib has a good effect on patients with AKT1E17K mutation and ER positive metastatic breast cancer [50]. Borussertib in combination with the MEK inhibitor trimetinib has shown antitumor activity in patient-derived xenograft models and provides a starting point for further pharmacokinetic/kinetic optimization [51]. In our study, two new highly selective inhibitors of AKT1 were screened: andropanoside (ZINC000049872065) and neoandrographolide (ZINC000021992902). However, these two drugs are not currently used as AKT1 inhibitors. Neoandrographolide directly binds to Rab5 by occupying the GDP/GTP binding channel to inhibit its function, highlighting the great potential of Neoandrographolide as a chemical therapeutic agent for cancer treatment [52]. Carbohydrate Modifications of Neoandrographolide for Improved Reactive Oxygen Species-Mediated Apoptosis through Mitochondrial Pathway in Colon Cancer [53]. Little research has been done on Andropanoside, existing studies mainly focus on their chemical structure and their cytotoxic effects toward LNCaP, HepG2, KB, MCF7, and sk-MEL2 human carcinoma cells and NO inhibitory effects in LPS-stimulated RAW264.7 cells [54]. Our study found that these two compounds have AKT1 inhibitory effects, providing the basis for the development of potential AKT1 inhibitors.

In summary, this study identified candidate compounds with inhibitory effects on AKT1 through a series of screening procedures, paving the way for clinical pharmacotherapy studies of AKT1 inhibitory drugs (such as the treatment of ovarian, lung, osteosarcoma, and pancreatic cancers). Finally, cell and specific inhibition experiments were conducted to verify the results of drug screening.

Although we have carefully designed all the details of the study, we must admit that there are still many shortcomings in our study. On the one hand, the safety of the drug still needs to be further considered, which requires more trials and more safety indicators, such as MTD (Maximum Tolerated Dosage) and AB (Aerobic Biodegradability). On the other hand, the selected compounds were not perfect. To improve their potential inhibitors, elaborate medication design, and refinement were needed in our future study.

## Conclusion

In order to screen and identify compounds that have targeted inhibitory effects on AKT1 from natural compound database ZINC15, a series of modules in Discovery Studio 4.5 were used in this study for step-by-step screening. Two compounds, ZINC000049872065 and ZINC000021992902, were predicted as potential inhibitors targeting AKT1. The experiments carried out by Discovery Studio 4.5 confirmed that these two compounds could bind tightly with AKT1 in the natural environments simulated by the MD simulation module. In addition, cell experiments confirmed the effectiveness of two compounds. This study lays the groundwork for future clinical trials of these two compounds. Moreover, these novel natural compounds with structural modifications can be potential contributors that lead to further rational drug design targeting AKT1.
